# A Study on Mobile Resources for Language Education of Preschool Children Based on Wireless Network Technology in Artificial Intelligence Context

**DOI:** 10.1155/2022/6206394

**Published:** 2022-06-07

**Authors:** QiuMing Li

**Affiliations:** Guangzhou Huashang Vocational College, Guangzhou, 511300 Guangdong, China

## Abstract

Preschool language education is a requirement of basic education reform as well as a requirement for children's growth in all aspects of body and mind. It is extremely important and valuable in encouraging the entire growth of preschool education as well as children's general harmonious development. The degree of informatization is changing day by day, and many information technology concepts and tools have entered the preschool education field. The Internet, electronic school bags, ECE whiteboards, terminal devices, and rich digital resources and tools have been introduced into kindergarten classrooms. The continuous advancement and application of information technology have provided the feasibility of building a smart learning environment for kindergartens. To this end, this paper starts from the core concepts and theoretical foundations of preschool education and sorts out the concepts of learning resources, smart learning, and smart learning environments. Learning theory, teaching theory, and activity theory provide the theoretical foundation for the creation of language learning tools in preschool education. The technologies of campus network, Internet of Things, artificial intelligence, and rich media are examined under the role and inspiration of smart learning environment to provide theoretical support for scientific design of smart language learning environment in preschool education.

## 1. Introduction

Today's society is developing rapidly, and in this era, the development and changes in the field of education have become a hot topic of concern [1]. To the dilemma faced by the reform of basic education at home and abroad, educational informatization has become an effective way out of the dilemma [2, 3]. The development of educational technology is a product of the combination of technological progress and educational development, and the concept of educational technology runs through the whole process of education, including, of course, preschool education [4–6]. The informatization of education has created more possibilities for learning [7]. The trend in modern preschool education is to build a wise learning environment in the early childhood learning environment, and this is one of the paths in the design of today's early childhood information-based learning environment [8]. Combining kindergarten curriculum goals and the needs of early childhood development, building a smart learning environment, and integrating mobile educational resources are the changes to the early childhood learning environment [9]. Kindergarten, as a crucial component of basic education, is intimately linked to the quality of learning that continues later and has a foundational role in the development of young children throughout their lives [10].

Language, as a vehicle for the individual's development, is of great importance for all aspects of human development [11]. As far as the individual is concerned, language is an essential tool for thinking, a form of cognitive ability, and an important sign of individual socialization. The preschool years are a period of rapid language development for young children, and the improvement of their language skills is gradually developed through constant communication and use [12]. Therefore, in the early childhood stage, which has a key impact on individual development, it becomes an issue that deserves our attention and in-depth research on how kindergartens can provide language education to children in a scientific and effective way during their natural growth process, so that children can acquire language skills and necessary communication skills in their life and learning [13].

Since the beginning of the twenty-first century, all walks of life around the world have proposed new-age goals and directions for the development of access to education [14]. As a result, smart learning environments have sprouted from the new era's requirements. Smart learning environments have become one of the core directions for the construction of learning environments. Since smart learning environments have been proposed, related research has sprung up, and the current stage is a critical period for exploration and construction. Most of the existing studies are on the application of smart learning environments in higher education, learning analytics in classrooms, and the application of Internet of Things technology in campuses [15–17]. Many modern information technologies have been developed to a more mature stage, but the application of modern information technologies in kindergartens and the study of smart learning environments in early childhood learning environments are sporadic [18]. Under the kindergarten wisdom learning environment, how to fully apply the existing technology to optimize the current kindergarten language learning environment, what level of kindergarten language education resources are actually available, and how to organically combine the information technology approach with the needs of the development of early childhood language education have become issues that need to be addressed urgently now.

To address this, we enhanced essential methodologies and characteristics of language education tools for young children based on their learning behavior characteristics, as well as their cognitive qualities and learning goals. We next examine and synthesize the data from the case studies in order to build an acceptable language learning programmer for early childhood preschool education. Explore the design of language education environments for young children based on the current state of their learning environments.

The paper's organization paragraph is as follows: The related work is presented in Section 2.  Section 3 analyzes the key technologies and features of educational environment for preschool children in wireless network environment.  Section 4 discusses the design of a kindergarten language education resource management system based on wireless network technology in an artificial intelligence environment. Finally, in Section 5, the research work is concluded.

## 2. Related Work

### 2.1. Current Status of Research on Information-Based Learning Environments in Preschool Education

The experimental study showed that teachers' use of whiteboards and electronic devices significantly improved children's literacy skills. Multimedia presentations create learning opportunities for children to interact tactilely with the whiteboard and also enrich the presentation of resources, giving children the opportunity to engage in multimedia dialogue and interaction [19]. Through data collection, methods used included observations, interviews, and a review of children's related documents to explore how early childhood educators can enhance young children's motivation to read through manipulating the classroom environment [20]. The study concluded that thematic reading and shared reading would enhance young children's motivation to read. There is a growing body of research showing that high-quality preschool environments improve child-teacher interactions and that teacher-student communication and interaction are very important aspects of learning activities. The computerization of the learning environment provides more possibilities for interaction between children and teachers, with real-time communication and off-site interaction becoming the norm. Information and communication technologies have limitations for the development of young children, but when properly designed and utilized, they will contribute to the intellectual, linguistic, social, and creative development of children ages 3-6.

In order to promote the healthy and harmonious development of children, the use of information technology in kindergartens should follow the three principles of simplicity, gamification, and appropriateness, and teachers should be proficient in designing and implementing information-based teaching activities [21]. At the same time kindergartens and relevant management departments should strengthen the common sharing of kindergarten information-based education and learning resources. Creating a good environment for children's games is an important means to play the educational function of games and environment [22]. The environment plays an important role in promoting the learning and play life of young children. By creating different levels of play environments, the basic educational tools of kindergartens can be realized. The introduction of multitouch virtual learning gadgets has aided in the optimization and improvement of technical tools, as well as creating a new situation of hands-on learning for young children with technical assistance. Virtual learning devices for young children are more attractive than traditional learning devices in terms of perceptual dimension, extended reuse, diversity, and state preservation.

### 2.2. Business Needs for Language Education Resources for Preschool Children

With the popularity of smart phones, the size of the mobile education market is at a rapid growth stage. The conclusion reached through continuous practical tests is that educational resources for preschool children need to be short, interesting, and educational. The business demand characteristics of auxiliary early childhood language education are shown in Table 1.

### 2.3. Student-Centered Teaching Theory

#### 2.3.1. Generative Teaching

Generative teaching emphasizes the subjectivity of students, and classroom ideas and teaching behaviors are adjusted according to the interactions and student responses in the classroom [23]. The characteristics of generative teaching are active student participation, nonpredetermined classroom, and interactivity. Generative teaching uses learning analytics to analyze and uncover dynamic learning paths and provide appropriate learning resources through data such as classroom learning records and online learning records of young children. Whether it is online learning, blended learning, or even traditional classrooms, as long as information technology exists, there is a need for learning analytics. The process of generative teaching and learning in a smart learning environment is shown in Figure 1.

#### 2.3.2. Effective Teaching

Effective teaching and learning theory assign three typical characteristics to classrooms: student-centeredness, focus on internal management, and commitment to instructional improvement [24]. The optimization of the learning environment is a strong guarantee for teaching improvement, and effective teaching needs the environment as support. Effective teaching is concerned with the measurability and quantification of learning outcomes. Quantitative learning outcomes provide dynamic adjustments to learning objectives and information, allowing for multiple levels of learning objectives to be provided based on student variability. An effective classroom learning environment requires the integration of three elements: pedagogy, technology, and social interaction. These three pedagogical elements correspond to three types of interactions: learner-content interaction, learner-other interaction (social interaction), and learner-operator interface interaction, as shown in Figure 2.

## 3. Key Technologies and Features of Educational Environment for Preschool Children in Wireless Network Environment

### 3.1. Key Technologies of Wireless Network Education Environment for Preschool Children

#### 3.1.1. Campus Network

As the link between kindergartens and the outside world, the campus network is the basis for the construction of the environment. The convenience and rapid development of the Internet have impacted the traditional learning style and educational philosophy of kindergartens. Big data-based analysis of students' online behavior preferences, network-based learning resources sharing, and cloud-based campus network webcast platform construction are all inseparable from the network as a medium of information transmission. The unified management technology of wired network and wireless network is applied to the campus network to solve the shortcomings that the wired and wireless cannot be managed uniformly in the past. The solution is shown in Figure 3. The BRAS (broadband remote access server) is a new form of access gateway for broadband network applications that is positioned at the edge layer of the backbone network and can complete data access of IP/ATM networks of user bandwidth, as shown in Figure 3.

#### 3.1.2. Internet of Things

IoT simply means connecting various objects through information and communication technology to form a connected and manipulee whole. With the characteristics of connectivity, human-object, and object-object union of wisdom, IoT plays a very important role in the smart learning environment. The purpose of IoT application in smart learning environment is sensing people and things and providing intelligent services. Intelligent sensing layer, information transfer layer, intelligent application support platform layer, and application layer are the four layers of the IoT structure.  Figure 4 depicts the architectural architecture of an IoT application on campus.

#### 3.1.3. Cloud Computing

The core idea of cloud computing is to manage and control a large number of network-connected computing resources to form a pool of computing resources that meet users' needs. Cloud computing is divided into three levels: cloud computing, cloud management, and cloud platform. The cloud computing platform is the key element to support the intelligent learning environment, and the intelligent learning environment based on cloud computing has three foundations. First, it supports the network infrastructure of the intelligent learning environment. The construction of the intelligent learning environment has a strong interconnection network, fiber optic network, remote backup storage network, centralized, secure, and high-speed network environment. At the same time, through the convergence of the three networks, the intelligent learning environment is provided with high-speed access to the cloud computing platform to ensure the safe and reliable operation of the intelligent learning environment network. Secondly, the cloud computing platform is the key element to support the intelligent learning environment. The cloud computing platform is the foundation to support the operation of the intelligent learning environment and provide huge services and resource management. It manages a large amount of highly virtualized computing, data, and resources generated by teachers and preschool children in the teaching process, forming a huge resource base and providing unified services. Third, the object-linked sensing system of the intelligent learning environment is the most common part of the overall intelligent learning environment operation and the most essential service level. Using FRID, sensors, collectors, QR codes, and ultrahigh definition camera monitoring devices and technologies, the intelligent management and safe, dynamic, real-time monitoring of the smart learning environment are realized.

#### 3.1.4. Augmented Reality

Augmented reality (AR) is a computer application, and human-computer interaction technology is developed on the basis of virtual reality technology, which presents users with a new environment combining reality and reality by fusing virtual information into the real environment. The three basic features of augmented reality are the fusion of real and virtual worlds, real-time interaction, and the precise alignment of virtual and real objects in 3D space. The application of augmented reality in learning refers to the fusion of a real or near-real 3D virtual situation constructed by a computer into a real situation, and the student enters and interacts with the situation by some means, thus building a reasonable understanding of the virtual situation and presenting a real scene. Learning in an augmented reality scenario includes four dimensions, namely, computer program, user, real world, and virtual environment, and the concept diagram is shown in Figure 5. Augmented reality originates in reality and returns to reality, and students interact with virtual situations with the aim of better understanding the real world. In the construction of intelligent learning environments for young children, augmented reality technology is used to enhance the authenticity and live feeling of learning situations. The vivid learning scenes help children understand the learning content more accurately and quickly, increase their interest in learning, and maintain a stable and positive learning mindset.

#### 3.1.5. Artificial Intelligence

Artificial intelligence technology has been widely applied in the sphere of education, thanks to the Internet's backing. Artificial intelligence has played a critical role in advancing smart education development. Providing the most effective intelligent learning support and services for learners is the goal of creating an intelligent learning environment. For example, in the development of intelligent question and answer system, intelligent learning system, and adaptive learning system, artificial intelligence technology needs to be combined with the Internet technology, multimedia technology, and big data technology. Through integration, they encourage each other to improve and expand one other's functions and application skills, so expanding and improving educational intelligence.

Currently, learning analytics technology analyzes the learning characteristics of learners using recorded data from the learning process in three forms: interactive text, video and audio, and system logs. Artificial intelligence algorithms can analyze quantitative metrics such as the number and percentage of online materials read and written by each learner and the number and percentage of messages that are responded to. It can also use social network analysis to calculate the centrality of each learner and perform cluster analysis of learners based on the information about the communication relationship between learners attached to the interactive text. The main content, the information on the classroom activity behavior of students and teachers, such as statistics on the frequency and proportion of children actively answering questions in class, the overall activity of the classroom, the proportion of questions asked, and the proportion of student discussions, is extracted through video and audio analysis. Automatic recognition of learners based on eye dynamics and body posture, conversion of learners' voice content into text content for analysis, and dynamic recognition of facial expressions, such as happy, sad, and angry, have all become possible thanks to the advancement of intelligent video and audio analysis technology. The use of gesture motions in the learning field improves the human-computer interaction experience significantly. In addition, the data index information established based on these analyzed data can greatly improve the efficiency and accuracy of summative and formative evaluations in teaching, such as statistics on classroom participation of specific children over a period of time, changes in children's emotions in the learning environment, and comparison of classroom performance of different learning contents.

### 3.2. Characteristics of Kindergarten Language Education Environment

The most fundamental aspect of an early childhood language learning environment is to reflect the “wisdom” of the learning environment. Smart kindergartens are kindergartens where new technologies are applied, where new technologies facilitate the kindergarten learning environment, and where the kindergarten learning environment is highly technologically oriented to achieve the integration of technology and the kindergarten. The design of smart learning environments for early childhood is a study of the application of technology, the development of kindergarten learning environments, and the design of smart kindergarten learning environments in the context of the use of new technologies. The integration of information technology with the characteristics of early childhood school environments has brought out more characteristics such as the playfulness and age-appropriateness of early childhood environments.

## 4. Design of a Kindergarten Language Education Resource Management System Based on Wireless Network Technology in an Artificial Intelligence Environment

After the previous analysis of the characteristics and technologies of the smart campus, we determined the architecture of the web-based preschool curriculum resource management information system with B/S mode, HTML+ASP technology in the foreground, and SQL SERVER 2019 in the background database.

### 4.1. Language Knowledge Module Tree Mind Map Design Structure

Examine the use of a tree route structure that resembles a mind map in the primary Chinese children's general knowledge modules. When compared to traditional structural system framework design ideas, it has numerous new advantages and features as part of the core framework architecture. This is particularly well suited to the dynamic embodiment of a user's thinking habits and the inner connection between knowledge points, which can realize the dynamic personality of the learning process for instant generation and is more in line with the constructivist concept of human-centered learning. Accordingly, the learning potential and learning needs also show obvious personalized characteristics. When using this module, there are several choice nodes on the learning path, and when reaching the nodes, different choices can form different learning paths, thus connecting the net-like learning resources through tree-like learning paths. Similar to the resource management structure of an interoperable highway network system, the learner is similar to a car driver driving on a highway network, whose choice of each turnoff determines the final route he or she will take.

This design structure is a cognitive structure for learning that best fits the natural attributes of children, changing the previous linear learning model in which learners passively receive learning content. Just like in the past, we could not choose the content of a movie; we could only decide to watch it or not; and once we bought a ticket, we had to enter on time. Later, we could choose the channel but not the content, and we could not jump back and forth. Later, with computers, you can select your own content, you can also play backwards and fast forward, and you can also have limited human-computer interaction, but there is no human-to-human communication. So there is the rapid development of the network, especially the popularity of instant messaging software such as WeChat, mobile portable chat software, and hardware represents the current trend of instant messaging interaction. The next step for wearable devices will eventually be to use wireless networks to connect people to people to form a true barrier-free interaction.

The nature of the thinking structure of the human brain's tree-like neuron mesh connection determines the technology's development in this direction, which means there is a logical isomorphism between the two, and the future will be towards the full depth of integration of the network management system and the human intelligent brain, i.e., embedded and wearable devices.  Figure 6 shows a tree mind map of the broad language knowledge modules for toddlers.

### 4.2. Literacy Module Design Structure for Preschoolers

Take the early childhood literacy module part as an example to explain the design function and operation process of specific functional modules. Login and registration for ordinary users: The early childhood literacy learning system implements member registration and login; first of all, you have to register in the entrance of this module; register a new user; click the Register Member button on the left side of the page to enter the member registration page; and only after successful registration, can you become an official user. Be sure to enter the correct email address when registering, so that you can get in touch with members in a timely manner. After logging in on the login page with the username and password of the administrator or regular user, you will enter this module. After logging into the early childhood literacy module, regular users can do the following: (1) browse the information in this section, as well as the knowledge of children's education; (2) view lessons and videos and browse pictures and animations; and (3) leave voice messages. The structure schematic is shown in Figure 7.

### 4.3. Learning Resources and Learning Activities in a Smart Learning Environment

For learning and teaching, the smart learning environment provides a large library of learning resources. Learning resources for young children include text, voice, animation, and tools, which are kept in the cloud and on the student's side. The smart learning environment provides a rich media environment for young children. According to the current learning situation and learning interests of young children, the smart learning environment designed in this paper will push out relevant resources.

Student information in the classroom is collected through cameras, and student data are automatically updated in the student attendance system. The face recognition platform can complete face detection and face recognition functions and realize the creation, modification, and query of face database. The smart learning environment uses video face recognition to establish the face database of the class of young children and completes face detection and recognition through the video data collected in the classroom. This function allows dynamic monitoring of students' attendance and departure from the classroom.

Augmented reality technology decreases the environmental modeling link and effectively increases the speed, flexibility, and fidelity of virtual 3D modeling by leveraging the perceptible, locatable, and operable human-computer interaction qualities of virtual reality. This also results in some new key technologies, such as display technology, three-dimensional registration technology, virtual and real lighting consistency technology, tracking registration technology, and natural interaction technology. First, the creation of the learning environment for young children should be integrated into the process of learning activities. Second, the virtual and real environment should be easy to build and disassemble to facilitate the efficient use of space. Third, use a variety of ways to mobilize children's overall perception and participation. Fourth, attention should be paid to meeting the individual learning and growth needs of young children. It is worth pointing out that augmented reality systems are a supplement to learning methods and cannot completely replace physical objects.

The smart learning environment offers a variety of language learning activities for young children, including audio-visual learning, cooperative learning, inquiry learning, and group learning. The learning tasks in semester education are divided into five categories: science, arts, social studies, language, and health. Children's language learning activities in the smart learning environment are shown in Figure 8.

## 5. Conclusion

Many information technology concepts and technologies have entered the field of preschool education as education informatization improves, and smart learning environments and smart campuses are becoming more widely recognized. The maturity and continuing growth of technology promote the continual progress of educational technology, from traditional classroom environments to multimedia classroom environments, and from multimedia classroom environments to virtual learning environments and smart learning environments. Although the research is at the level of theoretical assumptions and environment design, its educational significance and research value are worthy of recognition.

The development of wireless network technology and artificial intelligence has advanced the digital and intelligent transformation of traditional campus scenes. Using large-scale digital data within the new campus scenes can effectively improve the accuracy and universality of research results, which is a research hotspot in the field of learner analysis in the future. The core of this research includes exploring the key technologies and environmental features of language learning for preschool children in a wireless network environment relying on various technological tools, including artificial intelligence. The principles governing learning and teaching ideas and activities are used to create language learning resources and learning environments for young children. However, building a language learning resource environment for young children from the standpoint of a smart learning environment is insufficient; the research is locked at the level of design assumptions and lacks practical application consequences as support. Further validation of the environmental research design is needed in subsequent studies.

## Figures and Tables

**Figure 1:** Generative teaching generation process.

**Figure 2:** Interactive model of effective learning environments.

**Figure 3:** Integrated and flat campus network structure.

**Figure 4:** Structure diagram of IoT in smart kindergarten.

**Figure 5:** Augmented reality concept map.

**Figure 6:** Tree mind map of language knowledge modules for preschoolers.

**Figure 7:** Diagram of the structure of the early childhood literacy module.

**Figure 8:** Language learning activities in an intelligent learning resource environment for preschool children.

**Table 1:** Characteristics of business needs to support language instruction for young children.

1	Short and concise, able to tell a story, show a song, or complete a certain knowledge in a few minutes of scene presentation of a knowledge point
2	A combination of graphics, animation, and sound to enhance language learning for children
3	It takes up little space, is easy to transmit and store, and requires less hardware and equipment for teachers and institutions in weak clients.
4	You can find a wide variety of language works related to early childhood education materials or in line with teaching.

## Data Availability

The datasets used during the current study are available from the corresponding author on reasonable request.
